# The Value of CTA Based on Gold Nanorod Contrast Agent in Coronary Artery Diagnosis and Plaque Property Analysis

**DOI:** 10.1155/2021/5799133

**Published:** 2021-11-15

**Authors:** Heyu Bi, Liangshi Wang, Shupeng Wang, Qicheng Huang, Yue Sun

**Affiliations:** ^1^Department of Internal Medicine, Qiqihar Jianhua District Community Hospital, China; ^2^Center for Medical Imaging, The Third Hospital Affiliated Qiqihar Medical University, Qiqihar, 161000 Heilongjiang, China

## Abstract

Coronary CT angiography (CTA) with the characteristics of noninvasive and simple operation is widely used in the diagnosis of coronary artery stenosis. The choice of contrast agent exerts an important impact on the imaging quality of CTA. Conventional iodine contrast agents are easily excreted by the kidneys, from which the imaging window is short, and the imaging quality is poor. Metal nanomaterials have unique optical properties and have broad application prospects in imaging. Our aim is to explore the value of gold nanorod contrast agent in the diagnosis of coronary heart disease. A gold nanorod suspension was first prepared, and the prepared gold nanorod was uniform and had good dispersibility. It can be seen from the light absorption curve that there are two obvious peaks on the UV absorption peak of the gold nanorods. The gold nanorods were cultured in different solutions, and it was found that the particle size of the gold nanorods did not change significantly within 72 hours, indicating that the prepared gold nanorods had good stability. When observing the damage degree of mouse kidney tissue, it was shown that the damage degree of gold nanorod contrast agent to mouse kidney tissue was less than that of iodine contrast agent. The above results indicate that the gold nanorod contrast agent has good stability and safety. Therefore, our study demonstrated that the gold nanorod contrast agent has high value in the diagnosis of coronary arteries and the analysis of plaque properties.

## 1. Introduction

In recent years, due to more high-risk factors for cardiovascular disease, the incidence cardiovascular disease has continued to rise [1]. According to relevant epidemiological survey data, cardiovascular disease has become one of the main causes of human death, and the diseased population continues to be younger [2]. Coronary heart disease refers to the blood lipids depositing on the arterial intima due to abnormal body lipid metabolism, causing vascular lumen stenosis or occlusion, which leads to myocardial hypoxia, ischemia, or necrosis [3–5]. If the myocardial state can be accurately assessed in the early stages of coronary heart disease, targeted measures can be taken to reduce the risk of disability or death in patients. In addition, the current medical community believes that the nature of coronary artery plaque is closely related to the development of the disease. Therefore, analyzing the nature of coronary artery plaque in patients with coronary heart disease is of great significance for reducing the risk of cardiovascular disease.

CT is a method of scanning a predetermined layer of the human body through X-ray beams to obtain information and then obtaining reconstructed images through computer processing to examine the human body's pathological changes. However, when the patient has severely calcified vascular plaque, it will hinder the propagation of low-energy X-rays, resulting in distortion of the tissue CT value, which will result in ray hardening artifacts [6]. Coronary CT angiography (CTA), a noninvasive examination technique commonly used in imaging departments, is widely used in the diagnosis of vascular disease [7, 8].

The choice of contrast agent has an important impact on the imaging quality of CTA. At present, the largely used CT contrast agent in clinical practice is a small molecule iodine agent. However, the iodine contrast agent is easily excreted by the kidneys, resulting in a shortened imaging window, and its high osmotic pressure is easy to quickly balance inside and outside the blood vessel, reducing the imaging quality [9].

In recent years, the wide application of nanomaterials in medicine has provided new research directions for CT contrast agents. Compared with traditional small molecule contrast agents, nanoparticles have unique physical properties due to the adjustability of their size, shape, and composition. The nanoparticle-loaded contrast agents circulate in the blood for a longer time, and the renal clearance rate and capillary. The blood vessel permeability is low, which can enhance the imaging effect [10–14]. However, the development of nanoparticles in CTA imaging is still in its infancy. Since the first study of using gold nanoparticles as a contrast agent for CT scans in the early 20th century, researchers have successively modified gold nanoparticles with different functions, which makes gold nanoparticles have a wider range of uses [15]. The modified gold nanorods have good biocompatibility and safety, but they can circulate for a long time in the body and have broad application prospects in imaging [16].

Therefore, this study compares the value of traditional small-molecule iodine CT contrast agent and gold nanorod contrast agent in the diagnosis of coronary atherosclerosis plaque and the value of plaque character analysis, providing new information for the early diagnosis of coronary heart disease patients and the judgment of disease progression.

## 2. Materials and Methods

### 2.1. Main Reagents and Instruments

Thirty 6-week-old male ApoE knockout mice (ApoE-/-) without specific pathogens were provided by Beijing Huafukang Biotechnology Co., Ltd. (body weight 20.0 ± 0.5 g). Cetrimonium Bromide (CTAB) solution was provided by Dingguo Biotechnology Co., Ltd. The chloroauric acid solution was provided by the American Sigma Company. The sodium borohydride solution, sodium chloride solution, and chloroauric acid solution were all provided by Sinopharm Chemical Reagent Co., Ltd. Ascorbic acid was provided by Shanghai Macleans Biochemical Co., Ltd. Polyethylene glycol was provided by Ma Yinglong Pharmaceutical Group Co., Ltd. Micro-CT is provided by Siemens, Germany. The high-speed centrifuge is provided by Thermo Fisher Scientific Co., Ltd. Transmission electron microscopy and laser particle size analyzer were provided by Delong Company of the United States and Malvern Company of the United Kingdom, respectively.

### 2.2. Preparation of Gold Nanorod Contrast Agent

The gold nanorods are prepared first and then formulated into a suspension for use as a contrast agent. For synthesis and modification of gold nanorods, add 5 mL of cetrimonium bromide (CTAB) solution (concentration of 0.2 mol/L) to 5 mL of chloroauric acid solution (concentration of 0.0005 mol/L). Place the mixed solution in a 28°C water bath and stir gently. After the solution is fully mixed, slowly add 0.6 mL of ice-cold sodium borohydride solution (concentration of 0.01 mol/L) to obtain the gold seed solution. Add 25 mL of CTAB solution to a mixture of 750 *μ*L of silver nitrate solution (concentration of 0.004 mol/L) and 25 mL of chloroauric acid solution (concentration of 0.001 mol/L), and place it in a 28°C water bath and lightly stir gently until the solution is completely mixed. Finally, slowly add 350 *μ*L of ascorbic acid (concentration of 0.08 mol/L) to obtain growth fluid. Mix the gold seed solution (60 *μ*L) with the growth solution (50 mL), shake well, and let stand for 2 h to obtain the gold nanorod stock solution. Centrifuge the obtained stock solution (10000 r/min, 10 min), discard the supernatant, and place the concentrated gold nanorods in deionized water for resuspension. After 2 h of shaking, purified gold nanorods can be obtained. The purified gold nanorods were incubated with polyethylene glycol (PEG) at room temperature and centrifuged (10000 r/min, 15 min) after 1 h. The supernatant was discarded to obtain the PEGylated gold nanorods (the preparation process is shown in Figure 1). The obtained gold nanorods and water are prepared into a suspension with a concentration of 0.6 mg/mL for later use.

### 2.3. Characterization and Identification of Gold Nanorods

The gold nanorods prepared above were centrifuged (10000 r/min, 30 min) to remove excess CTAB, and the gold nanorods after centrifugation were transferred to a copper mesh and dried naturally at room temperature. A transmission electron microscope was used to observe the characterization of the dried gold nanorods, and an ultraviolet-visible spectrophotometer was used to detect its absorption spectrum.

### 2.4. Stability Analysis of Gold Nanorods

The gold nanorods were cultured in DMEM medium, sodium chloride solution (NS), and deionized water at room temperature, and the particle size changes of the gold nanorods at each time point were detected (the particle size distribution of the gold nanorods and the average particle size are detected by a laser particle size analyzer).

### 2.5. Scanning Method

After one week of adaptive feeding, 30 knockout mice were divided into regular group and nano group. Both groups were scanned by micro-CT. The contrast agent was injected into mice by tail vein injection. The regular group was injected with iopamidol contrast agent (23 mgl/mL, the injection rate was 0.5 mL/min), and the nano group was injected with gold nanorod contrast agent (0.7 mL/kg, the injection rate is 0.5 mL/min). Thirty minutes after the injection, the mouse was fixed in a special scanning catheter for enhanced scanning. The scanning parameters such as tube voltage (59 kV), tube current (167 *μ*A), and resolution (5 mm) were set and use 5 mm lead as a filter. For three-dimensional reconstruction, after scanning, use the NRecon software to synthesize one-dimensional and two-dimensional images into three-dimensional images. After reconstruction, use the CTvov software to model the acquired three-dimensional images, which is convenient for cutting and observing the coronary arteries of mice from various levels (transverse, sagittal, and coronal) (the scanning principle is shown in Figure 2).

### 2.6. Safety Analysis of Gold Nanorods

On the day after the scan, the kidney tissues of the two groups of mice were taken for HE staining, and the damage of renal tubular cells was analyzed. Take the mouse kidney tissue and cut it into 5 × 5 × 3 (cm) squares, and perform the steps of dehydration, paraffinization, embedding, sectioning, deparaffinization, and staining to obtain HE stained sections of the kidney tissue. Observe the pathological changes of the mouse kidneys under a light microscope (×200): 8 fields of view were randomly selected for each group, and the kidney damage of the mice was evaluated based on the expansion of the renal tubule lumen, blockage of the tube, flat cells, and cell necrosis and shedding. Set a total score of 1-5 points, where 1 point means no kidney damage, 2 points mean that the kidney damage is less than 1/5, 3 points mean that the renal tubule damage is between 1/5 and 1/2, 4 points indicate that the degree of renal tubular damage is more than 1/2, and 5 points indicate that all cells in the renal tubular have been damaged.

### 2.7. Image Quality Assessment

A 5-level scoring method was used to evaluate the imaging quality of all images. (1) For 1 point, the image has obvious artifacts, obvious noise, and no diagnostic value. (2) For 2 points, the image artifact is too large and accompanied by obvious noise, but the blood vessel edge structure is faintly visible. (3) For 3 points, the image artifacts are large, there is noise, and the blood vessel edge structure is blurred. (4) For 4 points, the image is relatively clear, there is a small amount of noise, and the blood vessel edge structure is relatively sharp. (5) The image is clear, the noise is small, and the blood vessel edge structure is sharp. Diagnosis can be made when the score is ≥3 points.

### 2.8. Statistical Analysis

In this study, the SPSS v.25.0 and GraphPad Prism v.8.0 software were used for data analysis. Quantitative data are expressed in the form of mean ± standard deviation, the comparison between the two groups is by *t*-test, and the comparison between multiple groups is by analysis of variance. The qualitative data is expressed in the form of *n* (%), and the chi-square test is performed. The comparison between all data is *P* < 0.05 indicating that the difference is greatly significant.

## 3. Results and Discussion

### 3.1. Characterization Analysis of Gold Nanorods

From the scanning image of the transmission electron microscope, it can be seen that the prepared gold nanorods have a uniform rod-like structure with good dispersibility, and the average long particle size is 30-40 nm (as shown in Figure 3(a)). It can be seen from the light absorption curve that there are two peaks on the UV absorption peak of the gold nanorods, at 500 nm and 690 nm, respectively (as shown in Figure 3(b)).

### 3.2. Stability of Gold Nanorods

It can be seen from Figure 4(a) that the particle size distribution of the gold nanorods prepared in this research is uniform and changes in a normal state. It can be seen from Figure 4(b) that the particle size of the gold nanorods did not change significantly within 72 h in deionized water, DMEM medium, and sodium chloride solution. The above results indicate that the gold nanorod contrast agent has good stability.

### 3.3. Safety of Gold Nanorods

Both iopamidol and gold nanorod contrast media are metabolized by the kidneys. Therefore, this study performed HE staining on mouse kidney tissue. After observation, it can be found that the kidney tissue of the mice in the regular group has obvious changes, mainly manifested as the obstruction of the renal tubule lumen, and the migration of renal tubule epithelial cells due to the accumulation of water in the lumen (as shown in Figures 5(a) and 5(b)). In the nano group, although renal tubules and glomeruli were also abnormal, the degree of abnormality was mild (as shown in Figures 5(c) and 5(d)). It can be seen from the score that the injury score of the regular group was 2.64 ± 0.31, which was greatly higher than that of the nano group 1.96 ± 0.28 (as shown in Figure 6 and Table 1). Therefore, we believe that gold nanorods as a contrast agent cause less damage to the kidneys of mice.

### 3.4. Comparison of Imaging Quality of Two Contrast Agents

After evaluating and comparing the imaging quality of the two groups of mice, it was found that the average imaging quality of mice using conventional iodine contrast agent was greatly lower than that of mice using gold nanorod contrast agent (as shown in Table 2 and Figure 7(a)). In addition, the imaging quality of all mice was analyzed, and it was found that the imaging quality of mice using conventional iodine contrast agents was concentrated at 3 points, while the imaging quality of mice using gold nanorod contrast agents was mostly 4 points (Figure 7(b)). Our data suggested that the gold nanorod contrast agent can improve the imaging quality of the coronary arteries in mice, presenting a higher value for disease diagnosis than traditional iodine contrast agents.

## 4. Discussion

Digital subtraction angiography is applied in assessing the degree and nature of vascular stenosis. However, the shortages including causing hematoma at the puncture site and generating a strong radiation limit its clinical application [17]. Compared with digital subtraction technology, CTA has been widely used in the diagnosis of coronary heart disease in recent years [18]. Based on spiral CT enhanced scanning, CTA used contrast agents and computational processing technology to reconstruct blood vessels into vascular images and then achieve the purpose of displaying vascular lesions [19]. The imaging quality of CTA is closely related to the types of contrast agents. At present, the most commonly used CTA contrast agents in clinical practice are small molecule iodine contrast agents (such as iodixanol, iopamidol, and iohexol). Mortezazadeh confirmed in vitro cell experiments that nanocontrast agents can improve MR imaging quality without increasing cytotoxicity [20]. Some other researches have stated that the signal-to-noise ratio of rhenium sulfide nanoparticle contrast agent is higher than that of iodine contrast agent, and the use of rhenium sulfide nanoparticle contrast agent in CT imaging can improve the contrast of gastrointestinal imaging in patients [21]. At present, the common CTA nanocontrast agents include nano suspensions, micelles, and nano latexes [22–24]. Metal nanoparticles have excellent quantum size effects, volume effects, and surface effects and are widely used in many fields such as catalysts, medical materials, and electromagnetic functional materials [25, 26]. In addition, due to their good biocompatibility, metal nanoparticles can exhibit plasmon resonance effects under visible light or infrared light [27]. Because of these properties, metal nanoparticles have broad application prospects in the preparation of contrast agents.

Gold nanorods are rod-shaped nanoparticles with unique optical properties that make them widely concerned in the field of biomedicine. They are often used in optical imaging contrast agents and tumor photothermal treatments [28–30]. In this study, a gold nanorod suspension was prepared, and its characterization, stability, and safety were determined. Through testing, it is found that the prepared gold nanorods present a uniform rod-like structure and have good dispersibility. It can be seen from the light absorption curve that there are two obvious peaks on the UV absorption peak of the gold nanorods. The gold nanorods were cultured in different solutions, and it was found that the particle size of the gold nanorods did not change significantly within 72 hours, indicating that the prepared gold nanorods had good stability. When observing the damage degree of mouse kidney tissue, it was found that the damage degree of gold nanorod contrast agent to mouse kidney tissue was less than that of iodine contrast agent. Our results indicate that the gold nanorod contrast agent has good stability and safety, highlighting that the gold nanorod contrast agent has high value in the diagnosis of coronary arteries and the analysis of plaque properties.

## 5. Conclusion

In summary, this study prepared a gold nanorod suspension and explored its value in CTA diagnosis of coronary heart disease. After identification, it was found that the prepared gold nanorods are uniform in size; have good dispersibility, stability, and safety; and can be used as a contrast agent for CTA. When comparing the imaging quality of gold nanorod contrast agent and conventional iodine contrast agent, it is found that the imaging quality of gold nanorod contrast agent for the diagnosis of coronary artery stenosis in mice is higher than that of conventional iodine contrast agent. Therefore, this study believes that the gold nanorod contrast agent has high value in the diagnosis of coronary arteries and the analysis of plaque properties.

## Figures and Tables

**Figure 1:** Flow chart of preparation of gold nanorods.

**Figure 2:** Micro-CT scanning principle diagram.

**Figure 3:** Characterization and analysis of gold nanorods: (a) transmission electron micrograph of gold nanorods; (b) absorption spectrum of gold nanorods.

**Figure 4:** Stability analysis of gold nanorods: (a) the particle size distribution of gold nanorods; (b) the change of the particle size of gold nanorods in different solutions.

**Figure 5:** The damage of different contrast agents to the kidneys of mice: (a, b) kidney tissue damage in mice using conventional iodine contrast agent; (c, d) kidney tissue damage in mice using gold nanorod contrast agent.

**Figure 6:** Comparison of kidney injury scores using different contrast medium groups.

**Figure 7:** Comparison of the imaging quality of the two contrast agents: (a) the average score of imaging quality of different contrast agents; (b) the score distribution of the imaging quality of the two contrast agents.

**Table 1:** Comparison of kidney damage in different contrast medium groups.

Grouping	Kidney injure score
Regular group	2.64 ± 0.31
Nano group	1.96 ± 0.28
*t*	6.305
*P*	<0.001

**Table 2:** Comparison of imaging quality using different contrast agent groups.

Grouping	Imaging quality
Regular group	3.91 ± 0.68
Nano group	3.34 ± 0.59
*t*	2.452
*P*	0.021

## Data Availability

All the raw data could be accessed by contacting the corresponding author if any qualified researcher need.
